# Antioxidant, Anti-inflammatory, and Antimicrobial Activity of the Kalanchoe pinnata and Piper longum Formulation Against Oral Pathogens

**DOI:** 10.7759/cureus.57824

**Published:** 2024-04-08

**Authors:** Jayasree Anandan, Rajeshkumar Shanmugam

**Affiliations:** 1 Nanobiomedicine Laboratory, Centre for Global Health Research, Saveetha Medical College and Hospital, Saveetha Institute of Medical and Technical Sciences, Saveetha University, Chennai, IND

**Keywords:** antimicrobial activity, biomedical applications, oral pathogens, piper longum, kalanchoe pinnata

## Abstract

Background

Dental caries stands out as a significant global infectious disease, with oral diseases posing substantial health concerns primarily due to bacterial, fungal, and yeast infections. *Kalanchoe pinnata* demonstrates antimicrobial, anticancer, antiparasitic, and hepatoprotective properties, with applications in various ailments. *Piper longum* exhibits potent antimicrobial effects against bacterial and viral pathogens due to the bioactive compounds within the plant. This study aims to assess the antimicrobial efficacy of *P. longum* and *K. pinnata* formulation against oral pathogens and evaluate its other biomedical potential.

Methodology

The agar well diffusion method was employed to assess the antimicrobial activity of the formulation containing *P. longum* and *K. pinnata* against oral pathogens. The protein leakage assay was employed to assess the ability of the prepared formulation to cause protein release from oral pathogens. The other biomedical potentials of the prepared formulation including cytotoxic effects, antioxidant, and anti-inflammatory properties were investigated using in vitro assays.

Results

The prepared *P. longum* and *K. pinnata* formulation demonstrated significant antimicrobial activity against tested oral pathogens, with inhibition zones observed for *Staphylococcus aureus* (32 mm), *Streptococcus mutans* (22 mm), and *Candida albicans* (12 mm). However, no inhibition was observed on *Enterococcus faecalis* at the highest concentration of 100 μL. Additionally, the formulation demonstrated significant antioxidant activity with percentages of 89.22%, 84.4%, and 86.93% in 2,2-diphenyl-1-picrylhydrazyl (DPPH), hydrogen peroxide (H_2_O_2_), and ferric (Fe^3+^)-reducing antioxidant power assays, respectively, at the maximum concentration of 50 μL. Furthermore, the formulation exhibited potential anti-inflammatory activity, as evidenced by 79% inhibition in bovine serum albumin (BSA) denaturation assay and 77% inhibition in egg albumin (EA) denaturation assay at the highest concentration of 50 μL. Additionally, the formulation displayed low cytotoxic effects, even at the highest concentration of 80 μL.

Conclusion

*K. pinnata* and *P. longum* formulation demonstrated potential antimicrobial efficacy against oral pathogens and exhibited diverse therapeutic potentials. Thus, the developed formulation could be used as a potential alternative for pharmaceutical drugs against oral pathogens.

## Introduction

The oral cavity serves as a complex microbial habitat within the human body, hosting a diverse variety of bacteria, yeast, and fungi. Although antibiotics have been used to treat various diseases, their indiscriminate use has led to the rise of multidrug-resistant pathogens [1]. Plants serve as valuable medicinal resources due to their potent antibacterial properties, proving highly effective in disease treatment [2]. Plants serve as valuable medicinal resources owing to their potential antibacterial properties, proving highly effective in the treatment of various diseases [3]. The significant potential of medicinal plants in developing new medications, capable of preventing or eliminating both spoilage and harmful bacteria, signifies their crucial role. In contrast to contemporary synthetic pharmaceuticals, natural remedies are more compatible with the human body [4].

*Kalanchoe pinnata* (*K. pinnata*), a succulent plant belonging to the *Crassulaceae* family, has been extensively utilized in traditional medicine for its anti-inflammatory, antidiabetic, and anticancer attributes [5,6]. Traditionally, it has been employed in ethnomedicine to various conditions such as burns, insect bites, peptic and gastric ulcers, abscesses, and inflammatory issues. Its applications in folk medicine extend up to acting as an astringent and analgesic as well as in the treatment of kidney stones and pulmonary infections [7].

*Piper longum* (*P. longum*), a flowering vine belonging to the family *Piperaceae*, is recognized for its diverse therapeutic applications, including respiratory tract infections, localized irritation, muscle discomfort, and inflammation [8,9]. Traditionally, *P. longum* has been utilized in medicine for conditions such as tuberculosis, cholera, chronic malaria, rheumatism, tumors, and spleen diseases. It also possesses antibacterial and antihepatocytic potentials [10]. The primary objective of the study was to investigate the antimicrobial capabilities of *K. pinnata* and *P. longum* against the oral pathogens and assess their biomedical potential through cytotoxic effects, antioxidant, and anti-inflammatory activities.

## Materials and methods

Preparation of plant formulation

The dried fruit of *P. longum *and leaves of *K. pinnata* were sourced from a local store located in Thiruverkadu, Chennai. Following collection, the plant parts were washed with double-distilled water to eliminate any undesired debris. Subsequently, 3 g each of *K. pinnata* and *P. longum *were combined with distilled water (100 mL) and subjected to boiling utilizing a heating mantle at 45°C for approximately 15 ± 2 minutes. The resulting formulation was subsequently filtered through Whatman filter paper grade No. 1 and condensed to 5 mL utilizing a heating mantle at 45°C. The condensed formulation was stored in a sealed container in the refrigerator for further use.

Antimicrobial activity

The antimicrobial activity of *K. pinnata *and *P. longum* formulation against oral cavity-causing pathogens, including *Enterococcus faecalis*,* Staphylococcus aureus*,* Candida albicans*, and *Streptococcus mutans*, was assessed using the agar well diffusion method. Various concentrations (25, 50, and 100 µL) of nanoparticles were tested, along with standard antibiotics amoxicillin (for bacterial culture) and fluconazole (for fungal culture). This assay followed the methodology outlined by Moghadam et al. [11].

Protein leakage analysis

The release of microbial proteins into the supernatant was employed to assess the integrity of microbial cells. Four microbial suspensions containing oral pathogens (*S. mutans*,* S. aureus*,* C. albicans*, and *E. faecalis*), each with a volume of 10 mL, were treated with varying concentrations of *K. pinnata *and *P. longum* formulation (25, 50, and 100 µL). Bacterial and fungal suspensions served as positive controls, while ampicillin (for bacteria) and fluconazole (for fungi) were used as standards. The assay followed the methodology outlined by Huang et al. [12].

Antioxidant activity

2,2-Diphenyl-1-Picrylhydrazyl (DPPH) Radical Scavenging Assay

The DPPH assay was employed to assess the free radical potential of the *K. pinnata *and *P. longum* formulation. The hydrogen bond transferring capability was determined by the decolorization of a methanol solution containing DPPH [13]. The antioxidant activity of various concentrations of the *K. pinnata* and *P. longum* formulation, along with standard ascorbic acid against DPPH free radicals, was determined using this assay. This assay followed the methodology outlined by Silva et al. [14]. 

*Hydrogen Peroxide (H_2_O_2_)* *Radical Scavenging Assay*

The H_2_0_2_ scavenging activity of the *K. pinnata* and *P. longum* formulation was assessed to explore its capability to neutralize H_2_0_2_ free radicals of various concentrations of the *K. pinnata* and *P. longum* formulation, along with standard ascorbic acid, was determined using this assay. This methodology followed the procedure outlined by Bhatti et al. [15].

Ferric Reducing Antioxidant Power (FRAP) Assay

The antioxidant activity of the *K. pinnata* and *P. longum *formulation was assessed by its ability to reduce ferric tripyridyltriazine (Fe^3+^-TPTZ) to ferrous tripyridyltriazine (Fe^2+^-TPTZ). Various concentrations of the *K. pinnata* and *P. longum* formulation, along with standard ascorbic acid, were tested for their capability to reduce Fe^3+^-TPTZ to Fe^2+^-TPTZ. This assay followed the methodology outlined by Guo et al. [16].

Anti-inflammatory activity

Bovine Serum Albumin (BSA) Assay

The anti-denaturation effect of the *K. pinnata* and *P. longum* formulation on BSA protein was assessed using the BSA assay. Additionally, the anti-inflammatory activity of the formulation at various concentrations (ranging from 10 to 50 µL) and diclofenac sodium was evaluated using this assay. The assay followed the methodology outlined by Kumar et al. [17].

*Egg Albumin (EA)* *Denaturation Assay*

The anti-denaturation effect of the *K. pinnata* and *P. longum* formulation on EA protein was assessed using the EA assay. Furthermore, the anti-inflammatory activity of various concentrations of the formulation (ranging from 10 to 50 µL) and diclofenac sodium standard was evaluated using this assay. The assay followed the methodology outlined by Chandra et al. [18].

Cytotoxic effect

The toxicology of the *K. pinnata* and *P. longum* formulation was assessed at various concentrations (5, 10, 20, 40, and 80 µL) and the sixth well was kept as a control (without adding formulation) in salt water. Each concentration was tested using ten nauplii and after 24 hours, and the percentage of live nauplii was calculated. This assay was conducted following the methodology outlined by Apu et al. [19].

## Results

Antimicrobial activity

Figure 1 shows the antimicrobial activity of the *K. pinnata* and *P. longum* formulation that was evaluated against the tested oral cavity-causing pathogens using the agar well diffusion method. In Figure 2, the graph depicts the potential antimicrobial activity of the prepared formulation against the tested organisms. At a concentration of 100 µL, the formulation exhibited maximum antimicrobial activity against *C. albicans* (12 mm), *S. aureus* (32 mm), *and S. mutans *(22 mm), with no inhibition for *E. faecalis*. However, compared to the standard amoxyrite, the prepared formulation demonstrated a slightly lower antimicrobial activity, except in *S. aureus*.

**Figure 1:** Antimicrobial activity of K. pinnata and P. longum against oral pathogens (a) E. faecalis, (b) C. albicans, (c) S. aureus, and (d) S. mutans *K. pinnata*:* Kalanchoe pinnata*; *P. longum*: *Piper longum*; *E. faecalis*: *Enterococcus faecalis*; *C. albicans*: *Candida albicans*; *S. aureus*: *Staphylococcus aureus*; *S. mutans*: *Streptococcus mutans.*

**Figure 2:** Graph representing antimicrobial activity of K. pinnata and P. longum against oral pathogens (a) E. faecalis, (b) C. albicans, (c) S. aureus, and (d) S. mutans *K. pinnata*:* Kalanchoe pinnata*;* P. longum*:* Piper longum*;* E. faecalis*:* Enterococcus faecalis*;* C. albicans*:* Candida albicans*;* S. aureus*:* Staphylococcus aureus*;* S. mutans*:* Streptococcus mutans.*

Protein leakage assay

Proteins are essential for the structural and functional integrity of bacterial and fungal cells. The effect of the *K. pinnata* and *P. longum* formulation on protein leakage from oral pathogens was investigated using this assay. As depicted in Figure 3, the results indicate that the prepared formulation induced protein leakage from the oral pathogens by disrupting the integrity of bacterial and fungal cells. In comparison to the protein leakage observed in the positive control, the leakage of proteins treated with the *K. pinnata* and *P. longum* formulation was higher at the maximum concentration of 100 µL. The results demonstrate that the protein leakage increases with the concentration of the formulation. Additionally, when compared to the standard amoxyrite, the prepared formulation exhibited lower protein leakage in *S. aureus, E. faecalis*, and *C. albicans*. However, in *S. mutans*, the prepared formulation induced more protein leakage.

**Figure 3:** Graph displaying the protein leakage analysis of the prepared K. pinnata and P. longum formulation (a) E. faecalis, (b) C. albicans, (c) S. aureus, and (d) S. mutans *K. pinnata*:* Kalanchoe pinnata*;* P. longum*:* Piper longum*;* E. faecalis*:* Enterococcus faecalis*;* C. albicans*:* Candida albicans*;* S. aureus*:* Staphylococcus aureus*;* S. mutans*:* Streptococcus mutans.*

Antioxidant activity

The antioxidant activity of the *K. pinnata* and *P. longum* formulation was evaluated using the FRAP, DPPH and H_2_O_2_ assays. In Figure 4a, the results of DPPH assay shows that at the lowest concentration (10 µL), the formulation exhibited a maximum inhibition of up to 61.37%, while at the highest concentration (50 µL), the inhibition reached up to 89.22%. Figure 4b illustrates the H_2_O_2_ free radical scavenging activity of the prepared formulation. The results demonstrate that at the lowest concentration (10 µL), the formulation displayed a maximum inhibition of up to 49.7%, whereas at the highest concentration (50 µL), the inhibition rose to 84.4%. Similarly, Figure 4c shows the FRAP assay of the prepared formulation. The results reveal that at the lowest concentration (10 µL), the formulation exhibited a maximum percentage inhibition at the highest concentration. Moreover, even at the lowest concentration, the formulation displayed potent inhibition against free radicals. The result indicates that when the concentration of the formulation increased, the percentage of antioxidant activity also increased.

**Figure 4:** Antioxidant activity of the K. pinnata and P. longum formulation using (a) DPPH assay, (b) H2O2 assay, and (c) FRAP assay *K. pinnata*:* Kalanchoe pinnata*;* P. longum*:* Piper longum.*

Anti-inflammatory activity

The *K. pinnata* and *P. longum* formulation was examined for its anti-inflammatory activity using the BSA and EA assays. The efficacy of the produced formulation to prevent the denaturation was evaluated through its anti-inflammatory activity. Figure 5a displays the BSA denaturation activity of the prepared formulation, and the results of the assay show that at the lowest concentration (10 µL), the formulation showed the maximum inhibition of up to 44%, and at the highest concentration (50 µL), the formulation showed the maximum inhibition of up to 79%. Figure 5b displays the EA denaturation activity of the prepared formulation, and the results of the assay show that at the lowest concentration (10 µL), the formulation showed the maximum inhibition of up to 51%, and at the highest concentration (50 µL), the formulation showed the maximum inhibition of up to 77%. The outcome of anti-inflammatory activity displays that the prepared formulation exhibits effects that are dose-dependent.

**Figure 5:** Graphs representing the anti-inflammatory activity of the K. pinnata and P. longum formulation using (a) BSA assay (b) EA assay *K. pinnata*:* Kalachoe pinnata*;* P. longum*:* Piper longum.*

Cytotoxic effect

The cytotoxic effect of the prepared *K. pinnata* and *P. longum* formulation was evaluated using the Brine Shrimp Lethality Assay (BSLA). Figure 6 displays the results of the cytotoxic effect, showing that the prepared formulation showed the low cytotoxic effect, even at the highest concentration of 80 µL by exhibiting 80% of live nauplii. At the lowest concentration of 5 and 10 µL, the formulation showed extremely low toxicity by exhibiting 100% of live nauplii. The results of the BSLA display the biocompatibility of the prepared formulation.

**Figure 6:** Graph dispaying the cytotoxic effect of the K. pinnata and P. longum formulation using the BSLA assay *K. pinnata*:* Kalanchoe pinnata*;* P. longum*:* Piper longum*;* *BSLA: Brine Shrimp Lethality Assay

## Discussion

The present study demonstrates that the prepared formulation of *K. pinnata* and *P. longum* exhibits potential antimicrobial activity, with a zone of inhibition on *S. aureus* (32 mm) and *S. mutans* (22 mm), followed by *C. albicans* (12 mm). However, the standard showed slightly higher antimicrobial activity compared to the prepared formulation. Furthermore, the prepared formulation induced significant protein leakage from all the oral pathogens, whereas the standard caused more protein leakage from all the pathogens except *S. mutans*. The prepared formulation showed potential antioxidant activity, exhibiting an 89.22% inhibition against DPPH radicals at 50 μL, 84.4% inhibition at the same concentration, and 86.93% in the FRAP assay. Nevertheless, the prepared formulation exhibited slightly less antioxidant activity in all the assays compared to the standard ascorbic acid. Additionally, the prepared formulation demonstrated potential anti-inflammatory activity, with a 79% inhibition on the BSA and a 77% inhibition on EA at the concentration of 50 μL. In the BSLA, 100% of live nauplii of brine shrimp at a concentration of 5 µL, and 80% were present at a concentration of 80 μL, indicating low toxicity and biocompatibility.

In a previous study, ethanolic extracts of *K. pinnata* demonstrated potential antibacterial activity against *C. albicans* and *S. aureus* [3]. Similarly, the crude extract of *P. longum* showed effectiveness against oral fungal pathogens, particularly for *C. albicans* [20]. Likewise, the prepared formulation in this study showed significant antimicrobial activity. Furthermore, the bioactive compound piperine present in *P. longum* displayed significant DPPH radical scavenging activity [21], while the extract of *K. pinnata* showed potent oxidative radical scavenging and antioxidant activity against DPPH free radicals [22]. Similarly, the prepared formulation exhibits excellent antioxidant activity in this study. Moreover, previous research has shown that methanolic crude extract of *K. pinnata* inhibits BSA denaturation in a dose-dependent manner [23], and silver nanoparticles prepared using *P. longum* exhibit potent anti-inflammatory activity [24]. Similarly, the prepared formulation displayed excellent anti-inflammatory activity in this study. Additionally, *P. longum* displays a potent cytotoxic effect on BSLA [25], while the crude extract of *K. pinnata* shows a low cytotoxic effect on brine shrimps [26]. Similarly, the prepared formulation displayed shows significantly less cytotoxic effect.

Limitations

In the present study, several in vitro analyses were conducted to evaluate the formulation. However, additional in vivo research, including animal and clinical trials, would be beneficial for a better understanding of its effects.

## Conclusions

The outcome of this study demonstrates the antimicrobial, antioxidant, anti-inflammatory, and cytotoxic effects of the crude formulation of *K. pinnata* and *P. longum*. The prepared formulation exhibits good antimicrobial activity against oral pathogens in the agar well diffusion method and induces the leakage of proteins in oral pathogens by damaging the bacterial and fungal cells in protein leakage assay. Additionally, the formulation acts as a free radical scavenging agent by inhibiting the DPPH and hydroxyl and by reducing the Fe^3+^-TPTZ complex to Fe^2+^-TPTZ. Through the inhibition of BSA and EA protein denaturation, it can also function as an anti-inflammatory drug. The formulation demonstrates an excellent cytotoxic effect, displaying the biocompatibility of the produced formulation. The results of the entire study indicate that the prepared formulation has potent antimicrobial and therapeutic applications, suggesting its potential use as a source for pharmaceutical drugs.
